# Application Analysis of 5G Intelligent Communication Technologies in the Field of Sports Distance Education

**DOI:** 10.1155/2022/2115041

**Published:** 2022-06-22

**Authors:** Yuanfeng Zhang, Majed

**Affiliations:** ^1^P. E. Scientific College, Harbin Normal University, Harbin, Heilongjiang, China; ^2^Tripoli Sports University, Tripoli, Libya

## Abstract

China has entered a new fifth-generation (5G) technological period, college students are relatively fast to absorb new things, and conventional teaching methods are incapable of properly stimulating students' interest in sporting activities. As a result, the 5G integrated teaching paradigm, which is based on communication technology, is an unavoidable reform of sports remote education. For a long time, technology and sports have been inextricably linked. However, new possibilities on the Internet are fast developing, resulting in massive volumes of data. In this paper, we propose a novel 5G framework for efficient sports distance education. Initially, the sports dataset is preprocessed using normalization, and the features are extracted using Principal Component Analysis (PCA). Following feature selection, a Hierarchical Multiscale Convolutional Neural Network (HM-CNN) is used to categorize and initialize the 5G utilizing the Enhanced Transfer Control Protocol (E-TCP) for efficient data transmission. The Elevated Ant Colony Optimization Algorithm improves the performance of the suggested system even more (EACO). The experimental results indicate that 5G integrated education reform based on communication technology may successfully enhance the number of college students' sports population.

## 1. Introduction

Education in China has grown increasingly computer-aided technology as a consequence of the country's fast educational informatization. The diversity of teaching approaches available to teachers now is more significant than in the past, and multimedia teaching formats have a variety of possible applications in the classroom. Teachers may make full use of “vision” to inspire students to think and learn new knowledge by using more flexible strategies of explaining and asking questions on the platform and utilizing more flexible techniques of explaining and asking questions. The study of human rhythmic movements is used to investigate various topics, including physical education, art, and performance. It is difficult to convey to language students the emotional meanings of sports and the rhythm of the accompaniment during the course of the education procedure. It is correct to say that the course materials properly depict the course content. The website has several images that motivate students to attain optimal cognition, are multimedia-rich, inspire excitement in studying, and help students to improve their knowledge and memory. In order to implement education on the network, it is impossible to utilize time, space, and other limits, and it is also impossible to use the network's capabilities to solve difficulties that arise.

From the aspect of activating students' learning ardor, physical education network teaching has the capacity to transform students from passive information receivers into active learners. Increasingly widespread usage of computers in the teaching profession has resulted from the growth of network multimedia technology and the improvement of the teaching environment inside educational institutions. It is intended to employ this rich and diverse carrier to communicate vital scientific information to students to boost students' comprehension and understanding using teaching strategies relevant to scientific knowledge. It has enabled even people who have not previously been able to make use of the Internet-based learning platform to now study sports whenever and wherever they desire. A greater number of educational resources may be shared across schools and sports fans as a result of this development. As a consequence of this growth, it is possible that a greater quantity of instructional materials will be shared across schools and sports enthusiasts. The timeliness, engagement, and presentation of multimedia networks make it feasible to bring sports learning into families and communities and any place with a network to allow more college students and nonschool sports enthusiasts to study online. However, as long as the use of several indices results in difficult operations and interference with duplicate information, it will be impossible to achieve the goal if the FPGA is used.

The possibility of reflecting data from the original indication is likewise available to it. It is estimated that the final figure will be based on the real-world 5G technology evaluation technique for evaluating instructors' teaching skills. An assessment technique such as this one may be used to analyze the final conclusion of the instructor and student performance evaluations, which can then be used to portray the teacher's direction in a somewhat objective way. We must consider both absolute and relative measurements while analyzing a situation. In order to limit the total assessment of a teacher's teaching of topic skills, Principal Component Analysis is employed in conjunction with other methods. The primary objective is to establish a traditional national sports educational resource platform in China, where educational resources are very inadequate. The purpose is to adhere to the resource integration approach of the traditional sports education resource platform while also satisfying the educational needs of learners from all over the world, regardless of time or region. This system can analyze and store information from the sports database at first, and then it can communicate educational material to the receiver using an Enhanced Transmission Control Protocol, which is a high-speed transmission protocol. In addition, we use raised ant colony optimization to optimize the transmission process while it is being transmitted.

According to studies on real-time data services, data communication is inextricably linked to real-time data gathering, real-time data management, and real-time data transmission. Delays or data loss may occur if communication protocols are not utilized correctly. As a consequence, selecting a suitable communication channel and protocol is critical. Other types of equipment are not needed for data collection since devices connected to the 5G Internet and the cloud computing center exchange data wirelessly. In order to overcome the aforementioned limitation, we propose a novel 5G architecture for an efficient sports distant education environment. In the beginning, the sports dataset is preprocessed using normalization, and then the features are extracted with the help of Principal Component Analysis (PCA). Following the selection of features, a Hierarchical Multiscale Convolutional Neural Network (HM-CNN) is used to classify and initialize the 5G network, which makes use of the Enhanced Transfer Control Protocol (E-TCP) for efficient data transfer and classification. The algorithm, known as the Elevated Ant Colony Optimization Algorithm, further increases the efficiency of the recommended system (EACO). In accordance with the trial findings, a 5G integrated education reform based on communication technology may be able to effectively increase the number of college students who participate in sports.

The rest of the paper can be organized as follows: Section 1 introduces the effectiveness of English teaching in improving network performance over information sharing. In contrast, the literature review on other existing methods is shown in Section 2.  Section 3 contains a problem statement, whereas Section 4 has a detailed discussion of the proposed amendment. The results in Section 5 illustrate that the proposed method is viable.

## 2. Related Works

The effectiveness of remote hybrid education and 5G, when combined with huge data collection and technology, will provide a more realistic learning experience for future learners, hence increasing the effectiveness of digital deep learning. As part of a bottom-up design and development technique for a 5G Open Class product, [1, 2] employed FIWARE middleware to manage all entities. They present a thorough architecture, technological platform, data formats, and end-user applications for 5G Open classes. They also demonstrate how to develop a cutting-edge location-based learning service. Wu et al. [3] discuss current improvements in energy-efficient wireless networks and how they could be applied to future next-generation cellular systems.

Following an examination of the trade-off between spectrum efficiency and energy efficiency, various research outcomes are discussed within a framework of energy-efficient resource allocation employing optimization as a common approach. Next, potential approaches for improving energy efficiency at the physical layer and during deployment are discussed. Other emerging technologies, such as massive multiple inputs and multiple outputs, device-to-device communications, and ultradense networks, have unsolved energy efficiency concerns, which have been emphasized as a consequence. Since VR technology has been used in many sectors in China, the authors of [4] demonstrated that the entrance of the 5G era provides a significant incentive for VR technology to take off again. The widespread adoption of 5G and virtual reality will greatly benefit higher education (VR). In light of the problems and inadequacies of current Chinese university landscape design teaching methods, such as the Introduction to Landscape Design course and teaching, Shah et al. [5] present 5G + VR technology to carry out the course system's unique design and teaching application. Feedback and evaluation of the teaching effect were completed. According to the findings of research and implementation, adding 5G + VR to landscape design instructional content and format simplifies and enlivens the learning experience for students while also creating a rich situational learning environment. A 5G cloud computing communication technique is used to assess changes in students' physical activity behavior and body composition before and after an experimental mix of instructional reforms and multimedia integration [6].

Smart cities and intelligent transportation systems will benefit from 5G technology [7]. It specifies the network class's important dimensions and features and the components of an intelligent city. Various smart city agility indicators will be examined to demonstrate the features of a smart city and what a smart city requires to be shared by 5G networks. In contrast to conventional towns, it is carried out in addition to online performance metrics and a few smart city activities [8]. Smart demands of savvy tourists, a tourist strip, and stakeholders will concentrate on greater performance. Smart tourism, resource optimization, and sustainable development have resulted in the creative use of technology to improve the quality of life in good governance and the tourist business. Yeu et al. [9] discuss current e-sports industry activities in China in terms of size, structure, and employment. With the comprehensive promotion and deployment of 5g technology, China's e-sports industry will accelerate the merger of offline and urban conventional industries with the support of local industrial policies, and China's e-sports sector will usher in a new round of industrial explosion cycle. Meanwhile, the e-sports business will focus its future research on e-sports game standards, 5G e-sports mode, professionalized e-sports sports, and e-sports education and culture. One of the objectives is to determine if technical, pedagogical knowledge levels and other variables are excellent predictors of how well distance education students will do in school [10]. The authors of [11] suggested a model-based approach to physical education, which incorporated a variety of diverse models for the first time. This study tackles the problematic difficulties head-on when it comes to developing, engaging with, and implementing a multimodal MBP idea. In general, MBP stresses the delivery of a model such as cooperative learning, physical education, social responsibility teaching, and understanding games. However, many studies have focused on how a single model is presented, whereas just a few have examined hybrid models that mix numerous models in a coherent and useable manner. Vasconcellos et al. look at the efficacy of self-determination theory in physical education. Using a multilevel structural equation modeling technique, they meta-analyzed data from 265 important papers obtained via considerable research. As predicted, self-motivation was favorably associated with desired goals and negatively associated with undesirable outcomes. As a consequence, the effects of intrinsic management are varied.

External control was inversely connected with adaptive results, although motivation was positively correlated with unpleasant outcomes. Instructors were shown to have a stronger impact on students' feelings of competence and autonomy than peers in the classroom, whereas connectivity in physical education was similarly related to teacher and peer effects. Renshaw et al. introduce the Constraints-Led Approach as a possible teaching option for sports and physical education instructors and academics (CLA). This strategy has since been implemented. Many academics have adjusted their attention to incorporate complexity as well as a more ecological perspective while utilizing the CLA style of teaching and coaching. When challenged with many constraints, the learner should self-organize in order to develop efficient movement options (task, environment, and performance). This, according to the CLA, is necessary. Wang et al. [12] created a physical education system that uses machine learning and IoT to detect athletic training qualities, forecast behaviors, and manage physical education and training data. Bringing artificial intelligence (AI) and the Internet of Things together (IoT), improvements have addressed a number of flaws in the original extreme learning machine to the hidden layer mapping and optimization techniques. Data is collected over time using Internet of Things technology, and after that data has been processed to a given degree, an extreme learning machine is utilized to anticipate the condition of sports training. The technology's effectiveness will be tested in the final trials. Based on the results, it seems that the proposed physical education and training system in this study may have real-world applications and might be used to enhance the current system. Gui et al. [13] investigated the use of virtual reality technology in physical education from a 5G standpoint.

Aerobics lessons are part of a college's general education curriculum. PE is used as an example in this research. They studied two freshmen classes, one as a control group and the other as an experimental group. The experimental class uses VRT to teach aerobics, while the control class uses traditional PE education as well as VRT to teach aerobics. Zhao et al. [14] look at the existing challenges in assessing university and college physical education instruction and the accompanying improved techniques. In order to improve the current assessment index system for physical education teaching in colleges and universities, the paper develops a new assessment index system for physical education based on multiple intelligence theory, taking into account teaching, teaching and learning, and management factors. Using fuzzy logic, the researchers in this work developed a complete method for grading college-level physical education training. The case study section exhibits the efficacy of this technique in attempting to assess physical education courses properly. Zeng et al. [15] evaluated the entire effect of PE education in colleges from the perspectives of instructors' teaching characteristics and students' learning impact using a hybrid technology of data mining and hidden Markov model. It begins by assessing the current state of college PE curriculum teaching quality assessment; then, it investigates the applicability of data mining technology and hidden Markov models to university PE teaching quality assessment and proposes a mathematical model for university PE teaching quality assessment; finally, it runs a series of tests based on mathematical models and thoroughly examines the results. The outcomes of the research indicate that the model presented in this work may increase the accuracy with which colleges assess the quality of physical education programs. The study's findings provide an informative look at how computer technology and language training might be combined. They provide a reference approach and an implementation methodology for machine learning technologies to improve collegiate physical education instruction. Wang et al. [16] discussed the use of virtual reality technology based on artificial intelligence in college PE training. The spline keyframe interpolation approach may be used to interpolate the position of the virtual human center of gravity, and the model posture formed in each frame is used to construct the virtual person's animations.

The animation may contain capabilities such as video storage, rapid playback, slow playback, and freeze after synthesizing three-dimensional human motion data. To clearly compare the participants' movements, virtual human animation and camera footage may be exhibited and played simultaneously on one display. Zhu et al. [17] showed that, because of its support and relevance, computing multimedia technology has a significant influence on the implementation of physical education reforms at universities and colleges. When it comes to university and college physical education reform and innovation, we should emphasize the value of computer multimedia teaching by emphasizing its advantages, developing a set of relevant work application concepts, and fully utilizing its benefits while also demonstrating its increased academic value in related teaching activities. Fan et al. [18] give a numerical assessment by comparing LTE's theoretical performance services to those provided by 5G, based on literature study and numerical evaluation results. Whether in K-12 or higher education, there is a continuing quest for improved methods to educate students. Because of the lower latency, 5G can accept (or delay) bigger volumes of data, which is beneficial for VR and other hyperrealistic support experiences. Support is given for embedded systems, language, and culture to provide an interface of building blocks needed by other developers. Sun et al. [19] investigate which 5G mobile networks are expected to experience traffic bursts and adapt to varying 5G deployment needs, as measured by the proposed Ultrareliable Low-Latency Communication (URLLC) algorithm being tested by different diverse research types' networks. The primary advantage of this system is the ability to execute a virtual network, in addition to 5G better transmission rates, decreased latency, remote execution, and a greater number of connected devices. For the deployment of 5G, Li et al. [20] use heterogeneous networks, notably for named data networking (NDN). NDN's future network architecture focuses on content to ease communications, with name-based forwarding conducted through the forwarding information base (FIB). This research provides an improved index known as a bitmap-mapping bloom filter as a unique FIB called B-MaFIB to increase the performance of NDN routers that can manage heterogeneous networks approaching 5G (B-MBF). Ma et al. [21] separate the output values of the long-term memory network from the hidden layer state values and vice versa. Incorporating an attention module into the brain's long-term and short-term memory networks boosts their output value and the value of their hidden layer state. Better and more accurate data classification was achieved by concentrating on the network's short- and long-term memory.

## 3. Problem Statement

Online education is fully dependent on wired Internet and mobile networks, imposing stringent requirements on network quality, software and hardware operating environment, and instructional facilities. As long as a bottleneck exists, it will negatively influence online teaching and may even prevent lessons from continuing. During the pandemic time, the enormous scale and large quantity of online teaching created a significant strain on the network environment, online teaching platform, and different network challenges. This happens every now and again. According to student questionnaire responses, the percentage of network impacting class reached 25%, ranking second in the amount of difficulties mentioned. The feedback reveals a variety of class issues, such as the inability to log in or connect to the Internet, video stuck, blurry video, no voice, and frequent connection loss. The major causes of these issues are low network quality and overcrowding on the online education platform.

## 4. Proposed Work

Beginning in 2020, the next generation of mobile Internet represented by 5G will be built and operated on a wide scale in China, considerably enhancing the quality of the mobile network environment on which online education is based. It can be predicted that, with the gradual promotion of the next-generation Internet of IPv6 and the gradual completion of 5G mobile Internet infrastructure, the network problems encountered by online teaching will gradually be solved, and the network environment of online teaching will greatly improve, over the next few years. While developing network infrastructure, we should encourage software and hardware development for online learning platforms.

We can also upgrade and optimize network servers and other facilities and types of equipment regularly, increasing the system's network concurrency limit and maximum data processing capacity and actively applying big data, cloud computing, artificial intelligence, VR/AR (Virtual Reality/Augmented Reality), and other advanced technologies to the online teaching platform to develop new functions and applications. The widespread use of these innovative new technologies will considerably extend the development area for online education and provide the groundwork for future online teaching.  Figure 1 shows a schematic illustration of the suggested technique.

### 4.1. Dataset

Every 5 minutes, eight people (four men and four women) participate in one of the 19 activities. Each subject's activity has a total signal length of 5 minutes. Because all of the activities were open-ended, participants were allowed to express themselves in whatever manner they saw fit. As a result, activity velocities and amplitudes varied amongst people. Data is captured at a sampling rate of 25 Hz using calibrated sensor modules. For each action, 480 (=60 × 8) signal segments may be created using a 5-minute signal.

The following are the 19 tasks:

- The act of sitting (A1)
- A position of strength and stability (A2)
- Sitting up straight and on the right side of the bed (A3 and A4)
- Taking the stairs up and down (A5 and A6)
- Taking a seat in an elevator without moving (A7)
- Taking a seat in an elevator (A8)
- Taking a stroll around a car park (A9)
- Walking at a pace of 4 km/h on a treadmill (flat and 15 deg inclined) (A10 and A11)
- Working out on a treadmill set at 8 mph (A12)
- Using a stair stepper to work out (A13)
- Using a cross-trainer for cardio exercise (A14)
- Alternating between horizontal and vertical positions when riding an exercise bike (A15 and A16)
- A rowing machine (A17)
- Bouncing (A18)
- Participating in basketball games (A19)

Because the information may be blended off, the physical information from the collected dataset can be categorized before it goes through the transmission process.

### 4.2. Preprocessing

Because the preprocessing process tries to eliminate undesired systematic variation in the data, we describe a method that uses variability to discover suitable normalizing factors. The observed data intensity variation may be used to compute the data variation as

(1) $$\begin{array}{c} X_{\text{ij}}=m_{i}\times y_{\text{ij}}\left(Z\right)\times e_{\text{ij}}, \end{array}$$

where *X*, *y*_*ij*_ represent the data intensity variations, *m*, *r*, and *e* represent the probabilistic constants, *i* and j represent the error factors, and *Z* represents the normalization factor.

(2) $$\begin{array}{c} Z=\log\;X,\Omega =\log\;Z,\mu =\log\;m,p\left(\Omega \right)=\log\;r\left(Z\right),\varepsilon =\log\;e,\\ Y_{\text{ij}}=\mu_{i}+p_{\text{ij}}\left(\Omega \right)+\varepsilon_{\text{ij}},\\ \varepsilon_{\text{ij}}∼N\left(o,\sigma_{i}^{2}\right). \end{array}$$

The randomness of the input error is as follows:

(3) $$\begin{array}{c} p_{\text{ij}}=\sum_{s}{µ}_{\text{is}}\left(\Omega_{\text{sj}}-\Omega_{s.}\right), \end{array}$$

where the average  *p*_ij_ is taken over the samples j = 1…M; that is, Ω_*s*._ ≡ 1/*M*∑_*j*_Ω_sj_. The parameters *µ* therefore relate the variability of internal standard intensities with the variability of intensities; that is, the bigger the parameter *µ*, the bigger the contribution of internal standard's *s* variability to the normalization correction factor of error peak *i*.

(4) $$\begin{array}{c} Y_{\text{ij}}∼N\left(\mu_{i}+p_{\text{ij}},\sigma_{i}^{2}\right),\\ =\sum_{j}\left(Y_{\text{ij}}-\mu_{i}\right)\left(\Omega_{\text{sj}}-\Omega_{s}\right)*\;\log\left(\underset{\text{ij}}{\prod }P\left(Y_{\text{ij}}|\mu_{i},p_{\text{ij}},\sigma_{i}^{2}\right)\right)=-\frac{1}{2}\sum_{\text{ij}}\left(\text{log}\left(2\pi \sigma_{i}^{2}\right)+\frac{{\left(Y_{\text{ij}}-\mu_{i}-\sum_{s}\beta_{\text{is}}\left(\Omega_{\text{sj}}-\Omega_{s}\right)\right)}^{2}}{\sigma_{i}^{2}}\right), \end{array}$$

where

(5) $$\begin{array}{c} \mu_{i}=\frac{1}{M}\sum_{j}Y_{\text{ij}}-\sum_{j,s}\left(\Omega_{\text{sj}}-\Omega_{s.}\right), \end{array}$$

(6) $$\begin{array}{c} \sigma_{i}^{2}=\frac{1}{M}\underset{j}{\sum }{\left(Y_{\text{ij}}-\mu_{i}-\sum_{s}\beta_{\text{is}}\left(\Omega_{\text{sj}}-\Omega_{s.}\right)\right)}^{2}. \end{array}$$

Since ∑_*j*_Ω_sj_ ≡ ∑_*j*_Ω_*s*_, (6) leads to

(7) $$\begin{array}{c} \mu_{i}=Y_{i}.*\;\Xi_{\text{is}}, \end{array}$$

where

(8) $$\begin{array}{c} \Xi_{is}=\underset{t}{\sum }\beta_{it}\sum ts. \end{array}$$

The equation can be rewritten as

(9) $$\begin{array}{c} \Xi_{\text{ts}}=\overset{\wedge }{\beta }\sum_{j}\left(\Omega_{\text{tj}}-\Omega_{t}\right)\left(\Omega_{\text{sj}}-\Omega_{s}\right),\\ \Xi_{\text{is}}=\overset{\wedge }{\beta }\sum_{j}\left(Y_{\text{ij}}-Y_{i}\right)\left(\Omega_{\text{sj}}-\Omega_{s}\right), \end{array}$$

where $\overset{\wedge }{\beta }$ is the error eliminating factor.

(10) $$\begin{array}{c} \overset{\wedge }{\beta }\equiv \overset{\wedge }{\Xi }\times \sum^{-1}. \end{array}$$

The hat matrix can be calculated by using the formula

(11) $$\begin{array}{c} {\tilde{X}}_{\text{ij}}=\overset{\wedge }{\beta }X_{\text{ij}}\times \;\exp-\sum_{s=1}^{s}{\overset{\wedge }{\beta }}_{\text{is}}\left(\Omega_{\text{sj}}-\Omega_{s.}\right),\\ {}*{\left(\frac{{\left(\prod_{k=1}^{M}Z_{1K}\right)}^{1/M}}{Z_{1j}}\right)}^{r_{i1}/\sigma_{i}^{2}}. \end{array}$$

The updated normalized function can be represented as

(12) $$\begin{array}{c} r_{i1}=\sigma_{i}^{2}\sum_{j=1}^{M}\left(\log\;X_{\text{ij}}-\log\;X_{i}\right)\left(\log\;Z_{1j}-\log\;z_{1}\right), \end{array}$$

where

(13) $$\begin{array}{c} \sigma_{i}^{2}=\sum_{j=1}^{M}{\left(\log\;Z_{1j}-\log\;z_{1}\right)}^{2}. \end{array}$$

### 4.3. Feature Extraction

Physical education covers a variety of topics. The characteristics may be derived based on the content. The PCA may be used to select features. The PCA may be used to derive statistical texture features of second order. Third- and higher-order textures, which make use of the interplay of three or more data pixels, have been used in a wide range of applications. The PCA, being an arithmetic function, frequently eliminates undesirable characteristics. It is simple to distinguish between specialized and undesirable traits. The data may be fanned out for analytical purposes. The frequency of data in a certain accurate differential area may be defined using PCA. In this scenario, the single-pointed feature will be examined, as well as undesired characteristics such as the l-feature and the unwanted detachment. When m returns a single value, it may be used to remove attributes from previously processed data. The process of dissociation may be as follows:

(14) $$\begin{array}{c} \text{Detachment}=D⊕V. \end{array}$$

To get the new value, we need to subtract the detachment value that can be illustrated as

(15) $$\begin{array}{c} E\theta A{=}_{A\left(i,j\right)}^{\wedge }\;\left[E\left(x+i,y+j\right)-B\left(i,j\right)+1\right],\\ -A_{\left(i,j\right)}\;\left[D\left(x+i,y+j\right)-B\left(i,j\right)-1\right]. \end{array}$$

After the process of the subtraction, the new eigencovariance matrix was obtained:

(16) $$\begin{array}{c} V_{N}\;V-\bar{V}=a_{1}u_{1}+a_{2}u_{2}+a_{3}u_{3}+\cdots +a_{N}u_{N}, \end{array}$$

where *V* represents the eigenvalues. The obtained symmetric feature matrix is in the form of

(17) $$\begin{array}{c} \overset{\wedge }{V}-\bar{V}=\sum_{i=0}^{1}a_{1}u_{1};\;1<N*d\left(a,b\right), \end{array}$$

where *d*(*a*, *b*)=∑_*i*=1_^*n*^*|*bi − ai. Finally, the subject-related features are selected.

### 4.4. Classification

Convolutional Neural Network (CNN) models are used to learn and categorize physical education information. Here, Multiscale Hierarchical CNN may be used to do categorization tasks. As a consequence of feature extraction, the instructional information must be divided into several games or work practices. This categorization was carried out using HM-CNN, a well-known approach. The aim is graded according to the probability that it will be achieved. It is a convolution algorithm that has already been trained. HM-CNN may be used to study a single dependent variable as well as one or more independent variables. Probabilities are calculated, and a function is applied using the HM-CNN. The information is gathered at the group level. HM-CNN can first read and resize the image before performing the classification procedure by determining the probability of its class. The smoother activation function may be computed for this purpose by using

(18) $$\begin{array}{c} g_{\text{Sact}}\left(y\right)=\frac{y}{1+e^{-\alpha y}},\\ \alpha \geq 0,g_{\text{Sact}},\\ \alpha ⟶\infty ,g_{\text{Sact}}, \end{array}$$

where *α* is the important parameter learned during the training process.

The extracted features can be converted into vectors for the process of the pooling,

(19) $$\begin{array}{c} B_{j}=\text{vec}\left(B_{j-1}\right)=\frac{1}{M\times M}\sum_{i=0}^{M\times M}F_{i},\\ B_{j}=\text{vec}=\text{af}\sum_{i=0}^{M\times M}w_{i}F_{i},\\ a=f_{\emptyset }\left(y\right),\\ f=a⊙\text{z,} \end{array}$$

where *a* is the pointed vectors and *f* is the specialized parameter.

Formally, the attention mechanism provides a neural network with the capacity to concentrate on a subset of the feature vectors by varying their weights accordingly. If we consider  *a*=*f*_∅_(*y*), *f*=*a*⊙z are the input vector, which can be a feature map, which can be an attention vector, and a network of attention with parameters can be illustrated as

(20) $$\begin{array}{c} B=-\frac{1}{n}\sum_{i=1}^{n}\sum_{k=1}^{C}1\left(z_{ik}=k\right)\ln\left(\frac{\exp\left({\left(w_{k}^{\text{out}}\right)}^{T}h_{k}^{\text{out}}\right)}{\sum_{j=1}^{C}\exp\left({\left(w_{j}^{\text{out}}\right)}^{T}h_{J}^{\text{out}}\right)}\right). \end{array}$$

This approach may be used to increase the accuracy and efficiency of a feature map in the HM-CNN model. Assume the input feature map is N by N, with C representing the size of the 2D map and C signifying the number of channels on the map. The attention module employs two consecutive convolutional layers to compress the feature map to a size of N-1 in the first stage. A locally connected 2D layer is then used to train N weights, which are subsequently activated using a sigmoid function. The weights are then repeated C times across the channel dimension using another convolutional layer. It is important to remember that this layer is followed by a linear activation function, which means that the weights might have a wide range of values. Nonetheless, after dividing the weight of the new feature map by the average weight vector, we scale the result by a factor of C. As a consequence, the final operation behaves similarly to a weighted average, with values that are in magnitude identical to the original feature vectors. Finally, the categorized weighted values may be expressed as

(21) $$\begin{array}{c} B=\gamma_{1}B_{1}+\gamma_{2}B_{2}. \end{array}$$

The equation can be rewritten as

(22) $$\begin{array}{c} B=\gamma_{1}\left(B_{1}+\frac{\gamma_{2}}{\gamma_{1}}B_{2}\right), \end{array}$$

where

(23) $$\begin{array}{c} \gamma =\frac{\gamma_{2}}{\gamma_{1}}. \end{array}$$

As a result of the classification, the different physical education subjects get classified. Then, it can be securely stored in the cloud for further transmission process.

### 4.5. 5G Network Deployment

A 5G wireless network design is being studied that randomly disperses and immobilizes all SN and some gateways. If the contact range of the sensor nodes is within the sensor nodes' range, sensor nodes will be allocated to each gateway. As a consequence, sensor nodes may be assigned to certain gates ahead of time. Because only a limited number of portals may be exchanged across sensor nodes, each needs its own list. The data gathering approach is divided into rounds, similar to the DSR research technique. Both SNs gather data from the surrounding environment throughout each cycle and transfer it to the relevant CH (i.e., the gateway). The data gates discard outdated and uncorrelated data before sending it to the base station through another CH acting as a next-hop relay node. The two nodes disconnect from the network after two rounds of turning off their power-saving communicators to conserve energy. Through the 5G wireless technology, everyone has access to the Internet. Despite such close proximity, the nodes are still wirelessly connected.

### 4.6. 5G Optimized Data Transmission

We recommend using optimized code to improve transmission quality since poor transmission quality of individual subflows may significantly impact the overall goodput of the Elevated Ant Colony Optimization-based Enhanced Transmission Control Protocol. Because it can dynamically vary its compression rate in response to receiving quality, the rate less optimal method beats fixed-rate compression. In this section, we will first go through the basic architecture of our proposed EACOBETCP. Data is encoded and delivered in several directions using the optimized code placed into the transport layer. The data allocation module is placed on top of the encoding module, which accepts a byte stream as input from the programs. Following that, each block is encoded, resulting in a series of encoded symbols being conveyed in packets and transmitted to the receiver. A decoding module is added to the data aggregation module to convert encoded symbols back to the original data on the receiver side. Decoded data may be provided to the application layer, and matched symbols can be deleted from the receiving buffer prior to transmission. When a transmission opportunity is received, the sender must generate encoded symbols from the waiting blocks and combine them into a packet for the subflow. After extracting the encoded symbols from the packets, the receiver will aggregate the symbols from separate subflows. The decoding module may utilize the received symbols if they are sufficient to recover a block. Using the Elevated Ant Colony Optimization Algorithm, we may begin the process of optimizing the TCP protocol's codes. The improved parameters for the ant colony optimization method are shown as follows:

(24) $$\begin{array}{c} A_{\min}=2*\sum_{i=1}^{n}{\text{AW}}_{i}*\max_{1\leq i\leq n}{\text{RTT}}_{i}. \end{array}$$

The optimized parameters for the Elevated Ant Colony Optimization Algorithm can be illustrated as

(25) $$\begin{array}{c} {\text{EA}}_{\min}=\sum_{i=1}^{n}{\text{AW}}_{i}*\left(\max_{1\leq i\leq n}{\text{RTT}}_{i}+\max_{1\leq i\leq n}{\text{RTO}}_{i}\right). \end{array}$$

By using the elevated parameters, the buffer size for the sender and the receiver can be minimized by using the following equation:

(26) $$\begin{array}{c} d_{n}=\left(\sum_{k=1}^{{\overset{\wedge }{k}}_{a}}q_{k}.g_{\text{nk}}\right)\mathrm{mod}2, \end{array}$$

where $n=\text{by}-{\overset{\wedge }{k}}_{a}{\left(g_{\text{nk}}\right)}^{\prime }s$.

In our proposed protocol, we used some optimized codes which are rate less, which was based on the EACO that can be represented as

(27) $$\begin{array}{c} \partial_{a}\left(l_{a}\right)=\sum_{j>l_{a}}\left(\begin{array}{c} {\overset{\wedge }{w}}_{f}+l_{a}\\ j \end{array}\right)q_{f}^{i}{\left(1-q_{f}\right)}^{{\overset{\wedge }{w}}_{f}+l_{a}-j}. \end{array}$$

The probability of the coding failure can be illustrated as

(28) $$\begin{array}{c} P=q_{f}^{j}{\left(1-q_{f}\right)}^{{\overset{\wedge }{w}}_{f}+l_{a}-j}. \end{array}$$

where $q_{f}=\left(\begin{array}{c} {\overset{\wedge }{w}}_{f}+l_{a}\\ j \end{array}\right)p_{f}^{j}{\left(1-q_{f}\right)}^{{\overset{\wedge }{w}}_{f}+l_{a}-j}$.

(29) $$\begin{array}{c} j>l_{a},\\ p_{f}=\frac{{\overset{\wedge }{k}}_{a}+l_{a}}{k_{a}}. \end{array}$$

The probability of the packet loss can be defined by using the following equation

(30) $$\begin{array}{c} {\text{EDT}}_{f}=\sum_{j=0}^{\infty }q_{f}^{j}\left(1-q_{f}\right){\text{jRTO}}_{f}+{\text{DT}}_{f}\\ =\frac{q_{f}{\text{RTO}}_{f}}{1-q_{f}}+{\text{DTf}}^{*}. \end{array}$$

The expected arriving time of the packet (RTT_*f*_) can be demonstrated as

(31) $$\begin{array}{c} {\text{RTT}}_{f}=\left(1-q_{f}\right){\text{RTT}}_{f}+q_{f}{\text{RTO}}_{f}. \end{array}$$

The subflow for the packet can be calculated step by step:

(32) $$\begin{array}{c} {\text{EAT}}_{f}=\left\{\begin{array}{c} {\text{EDT}}_{f},\text{if }w_{f}>0\\ {\text{EDT}}_{f}+{\text{RT}}_{f}-T_{f},\text{otherwise } \end{array}\right.,\\ {\text{EAT}}_{f}={\text{EDT}}_{k}+{\text{ RT}}_{k}-T_{k}<{\text{EAT}}_{j},\\ {\text{EDT}}_{1<}{\text{EDT}}_{2<\cdots \cdot <}{\text{EDT}}_{n+1},\\ {\text{PEDT}}_{2<}{\text{PEDT}}_{3<\cdots \cdot <}{\text{PEDT}}_{n+1},\\ {\text{PEDT}}_{1}=\left(1-q_{2}\right)\frac{r_{2}}{2}+q_{2}\left(R_{2}+{\text{EDT}}_{1}\right),\\ =\left(1-q_{2}\right)\left(\frac{r_{2}}{2}+\frac{q_{2}R_{2}}{1-q_{2}}\right)+q_{2}\left(R_{2}+{\text{EDT}}_{1}\right)\\ =\left(1-q_{2}\right){\text{EDT}}_{2}+q_{2}{\text{EDT}}_{1},\\ {\text{PEDT}}_{2}>{\text{EDT}}_{1},\\ {\text{PEDT}}_{1}<{\text{PEDT}}_{2},\\ \frac{{\text{EDT}}_{2}}{{\text{EDT}}_{1}},\\ m>\frac{3-q_{1}}{1+q_{1}},\\ {\text{PEDT}}_{2}=\frac{q_{2}R_{2}}{1-q_{2}}+\frac{r_{2}}{2}\approx \frac{1+q_{2}}{2\left(1-q_{2}\right)}r_{2},\\ {\text{EAT}}_{1}<{\text{EDT}}_{1}+{\text{RT}}_{1}-T_{1},\\ <{\text{EDT}}_{1}+R_{1},\\ \approx \frac{{\text{EDT}}_{2}}{m}+r_{1},\\ {\text{EAT}}_{f}<{\text{PEDT}}_{2}. \end{array}$$

The optimized subflow can be calculated as follows:

(33) $$\begin{array}{c} \frac{E\left(T_{2}\right)}{\;E\left(T_{1}\right)}\leq q_{2}\frac{3-q_{1}}{1+q_{1}}+\left(1-q_{2}\right)m. \end{array}$$

Then finally, the best fitness path can be identified by using the following equation:

(34) $$\begin{array}{c} E\left(T_{2}\right)=\left(1-q_{2}\right)\frac{r_{2}}{2}+q_{2}\left(R_{2}+E\left(T_{1}\right)+E\left(RT_{1}-T_{1}\right)\right),\\ \leq \left(1-q_{2}\right)\frac{r_{2}}{2}+q_{2}\left(R_{2}+E\left(T_{1}\right)+R_{1}\right),\\ E\left(T_{2}\right)=m=\frac{{\text{PEDT}}_{2}}{{\text{PEDT}}_{1}}\approx \frac{\left(1+q_{2}\right)\left(1-q_{1}\right)r_{2}}{\left(1-q_{1}\right)\left(1-q_{2}\right)r_{1}}. \end{array}$$

The elected optimized path transmission process can be represented as

(35) $$\begin{array}{c} E_{\text{TX}}\left(k,c\right)=E_{\text{elec}}*k+\epsilon_{\text{OPT}}*k*d^{2\;}\text{ if }d<d_{0},\\ E_{\text{elec}}*k+\epsilon_{\text{OPT}}*k*d^{4\;}\text{ if }d\geq d_{0},\\ E_{\text{RX}}\left(k\right)=E_{\text{elec}}*k. \end{array}$$

Finally, the data can be securely transmitted within a limited period of time.

## 5. Performance Analysis

This section illustrates the efficacy of the proposed approach. Many online education apps are large in capacity, yet they may support hidden antijamming wireless networks. They perform an important purpose, and subsequent orders will not need the same high data rate connections. The suggested technique has two major features: low-latency communication and ultrareliable communication. 5G can provide up to 20 gigabits per second of data speed and a peak data throughput of 100 megabits per second (Gbps). While average and peak data speeds for 4G are also 100 megabits per second, this is light years ahead of that (gbp). In order to improve the platform's scalability, it is recommended in this research that a new data packet processing architecture be constructed based on a combined simulation scheme of optimization technologies (Table 1).

In this case, the input data may be preprocessed and categorized based on the retrieved characteristics. The HCNN approach was used to categorize the physical education materials. The proposed classifier's performance may be evaluated by comparing it to several current techniques [21]. This paper uses six metrics to assess the overall effectiveness of the classifier model: accuracy, recall, F1 score, ROC, and AUC. Deep learning algorithms have long depended on these indicators to assess their performance. This study includes a more detailed classification effect expression to assist readers in better understanding the results. The mathematical equation for the given index is provided as follows:

(36) $$\begin{array}{c} \text{Accuracy}=\frac{\text{True Positive}+\text{True Negative}}{\begin{array}{c} \text{True Positive}+\text{False Negative}+\text{False Positive }\\ +\text{True Negative} \end{array}}\text{,}\\ \text{Precision}=\frac{\text{True Positive}}{\text{True Positive}+\text{False Positive}}\text{,}\\ \text{Recall}=\frac{\text{True Positive}}{\text{True Positive}+\text{False Negative}}\text{,}\\ F_{1}=\frac{2*\text{Precision}*\text{Recall}}{\text{Precision}+\text{Recall}}.\\ \text{TPR}=\frac{\text{True Positive}}{\text{True Positive}+\text{False Negative}}.\\ \text{FPR}=\frac{\text{False Postive}}{\text{False Positive}+\text{True Negative}}. \end{array}$$

Figure 2 depicts the proposed classification technique, which has a maximum accuracy yield of 99.8%, which is much higher than that of traditional classification methods.

Figure 3 illustrates the proposed classification approach, which achieves a maximum accuracy yield of 98 percent, which is much higher than that of standard classification methods.

A maximum memory yield of 98% is shown in Figure 4, making it superior to traditional categorization techniques in terms of recall yield. References [18, 19] and [20] may be used to demonstrate the effectiveness of the proposed 5G optimized TCP network data transmission technique in comparison to certain other current approaches to demonstrate efficiency.

However, the attack surface will be significantly increased because of the large number of linked devices and the usage of network virtualization technologies in the core infrastructure. If a single error or malicious software brings down the whole network, the entire civilization is placed in danger. As seen in the following graph, the data transmission efficiency of 5G is much greater than that of 4G. In a nutshell, the demonstration's goal is to demonstrate how flexible 5G network and infrastructure scheduling can be accomplished. The suggested strategy has a success rate of 90% in most cases. DND and LLCUR produce 72% and 85%, respectively, in the preceding methods (Figure 5).

It is observed that, when compared to another approach, the 5G optimized TCP methodology has lower latency throughout the network (Figure 6).

The outcomes of a study on temporal complexity are shown in Figure 7. When the suggested procedure is completed, it takes 38 milliseconds. Using current methodologies, Data Named Design (DND) (LLCUR) yields 42 ms and 44 ms, respectively. The suggested system requires less time to implement than other similar systems now in use.  Table 2 shows the overall performance of the proposed 5G system in terms of data throughput.

Figure 8 depicts the performance of the proposed network when it comes to data transmission and storage. Compared to other current approaches, a greater variety of data transmission speeds is available with the proposed protocol.

On the other hand, Figure 9 depicts the performance of the proposed network in terms of data transmission security. A wide variety of data transmission security rates is available with the suggested protocol, which is more than that available with other standard approaches.

It is obvious from Figure 10 that the current physical education platform does not meet the needs of a large number of people, especially the general public. For this reason, as expected, the debut of 5G platforms will be incredibly valuable due to the sluggishness, inefficiency, and time-consuming nature of network data transfer. As a result, the satisfaction rate was almost equal to the anticipation rate while using the 5G technique that was proposed. In order to provide a better future for the communication and data transmission infrastructure, the proposed 5G optimized ETP should be implemented.

The performance analysis of each network is shown in Figure 11; (a) depicts the execution up to the goal normal bit rate, and (b) depicts a schematic depicting the exchange of records lasting one megabyte in duration. Even if the touch rate is 720, which is sent as a level of the spot rate required by the 100 clients, the touch rate is only 1080 and 4 K. At any rate, one message is 83 bytes long. Also, the client aim of another of the observed piece rates relates to the fact that the obtained competitor was lower than expected, but that not all of the information was obtained. These are the consequences; with the above-depicted accentuation serving as an example, there is a goal to information misery, and it is to harm people.

## 6. Conclusion

This paper demonstrates that most people are looking forward to the debut of the 5G physical education information platform design. A 5G network is being used to develop online contact for basketball teaching purposes. As mobile communications capacity rises, the 5G network will take off and become unavoidable. These speed up data transmission and open up a whole new world of commercial and educational opportunities. In addition, using a 5G network for low-latency communication has a favorable influence on daily life. 5G will have a variety of distinct qualities, including the capacity to swiftly deploy services and management algorithms, function autonomously, and make better use of resources during online training. Because there were few similar systems available for comparison and because users' expectations and process linkages were not clearly defined, developing educational information system requirements took just a short period from idea to implementation. When adopting the proposed technique, network speed is 98%, data transfer efficiency is 90%, and time complexity is 38%.

## Figures and Tables

**Figure 1:** Schematic representation of the suggested methodology.

**Figure 2:** 5G data versus accuracy.

**Figure 3:** 5G data versus precision.

**Figure 4:** 5G data versus recall.

**Figure 5:** Number of files versus efficiency.

**Figure 6:** Time versus latency.

**Figure 7:** Number of files versus time complexity.

**Figure 8:** Network size versus performance.

**Figure 9:** Network size versus security.

**Figure 10:** Suggested 5G performance and satisfaction analysis.

**Figure 11:** Performance of each network.

**Algorithm 1:** EACOBETCP.

**Table 1:** Simulation specifications of the suggested system.

Parameters	Values
Energy transmission	100 m
Energy sampling	20
Energy amplitude	0.0128 m
Energy aggregate	8 kWh
Number of packets	Random of 15–20
Square area size	1000 ^∗^ 1000 m^2^
Velocity	[15, 40] m/s

**Table 2:** Performance of the suggested data transmission.

Number of terminals	Number of successful packets	Packets transmission success rate (%)	Simulation run time
10	1000	100	13.6
50	2000	99.8	25
100	3500	89.9	61.7
500	5000	85.5	85.5
1000	5500	78.6	120
5000	5200	68.5	248

## Data Availability

The datasets used during the current study are available from the corresponding author upon reasonable request.
